The article "The Role of Thymosin Beta 4 on Odontogenic Differentiation in Human Dental Pulp Cells" was retracted in 2025. Reasons: duplicated images; duplicated data; duplicate publication; overlap with earlier publications.

# The Role of Thymosin Beta 4 on Odontogenic Differentiation in Human Dental Pulp Cells

**DOI:** 10.1371/journal.pone.0061960

**Published:** 2013-04-17

**Authors:** Sang-Im Lee, Duck-Su Kim, Hwa-Jeong Lee, Hee-Jae Cha, Eun-Cheol Kim

**Affiliations:** 1 Department of Maxillofacial Tissue Regeneration, School of Dentistry and Institute of Oral Biology, School of Dentistry, Kyung Hee University, Seoul, Republic of Korea; 2 Department of Conservative Dentistry, School of Dentistry, Kyung Hee University, Seoul, Republic of Korea; 3 Department of Parasitology and Genetic, Kosin University College of Medicine, Busan, Republic of Korea; Instituto Butantan, Brazil

## Abstract

We recently reported that overexpression of thymosin beta-4 (Tβ4) in transgenic mice promotes abnormal hair growth and tooth development, but the role of Tβ4 in dental pulp regeneration was not completely understood. The aim of this study was to investigate the role of Tβ4 on odontoblastic differentiation and the underlying mechanism regulating pulp regeneration in human dental pulp cells (HDPCs). Our results demonstrate that mRNA and protein expression of Tβ4 is upregulated during odontogenic differentiation in HDPCs. Transfection with Tβ4 siRNA decreases OM-induced odontoblastic differentiation by decreasing alkaline phosphatase (ALP) activity, mRNA expression of differentiation markers, and calcium nodule formation. In contrast, Tβ4 activation with a Tβ4 peptide promotes these processes by enhancing the phosphorylation of p38, JNK, and ERK mitogen-activated protein kinases (MAPKs), bone morphogenetic protein (BMP) 2, BMP4, phosphorylation of Smad1/5/8 and Smad2/3, and expression of transcriptional factors such as Runx2 and Osterix, which were blocked by the BMP inhibitor noggin. The expression of integrin receptors α1, α2, α3, and β1 and downstream signaling molecules including phosphorylated focal adhesion kinase (p-FAK), p-paxillin, and integrin-linked kinase (ILK) were increased by Tβ4 peptide in HDPCs. ILK siRNA blocked Tβ4-induced odontoblastic differentiation and activation of the BMP and MAPK transcription factor pathways in HDPCs. In conclusion, this study demonstrates for the first time that Tβ4 plays a key role in odontoblastic differentiation of HDPCs and activation of Tβ4 could provide a novel mechanism for regenerative endodontics.

## Introduction

Dental pulp has the capacity to generate reparative dentin in response to damage from infection, exposure, trauma, and chemicals [1]. Reparative dentinogenesis requires the growth and differentiation of dental pulp cells (DPCs) into odontoblasts [2]. The mineral formation process during dentinogenesis appears to involve highly controlled expression of non-collagenous proteins secreted primarily by odontoblasts, such as osteonectin (ON), osteocalcin (OCN), osteopontin (OPN), bone sialoprotein (BSP), dentin matrix protein-1 (DMP-1), and dentin sialophosphoprotein (DSPP) [3], [4]. Thus, the regulation of odontogenic differentiation in human DPCs (HDPCs) has important implications for the development of new therapeutic strategies for vital pulp therapy, but the molecular mechanisms inducing odontoblastic growth and differentiation remain to be elucidated.

Thymosin beta-4 (Tβ4) is a 4.9-kDa actin sequestering peptide, which binds to monomeric globular actin and inhibits actin polymerization [5]. Tβ4 has multiple biological activities, including promotion of angiogenesis [6], [7], chemotaxis [8], inhibition of inflammation, and wound healing [9]. Tβ4 is upregulated during endothelial cell differentiation and has been shown to stimulate angiogenesis by differentiation and directional migration of endothelial cells and tube formation [10]. Furthermore, Tβ4 has been shown in various rodent models to promote stem cell migration and differentiation into keratinocytes and hair follicles in the bulge region, inducing dermal repair and causing increased hair growth [8], [11].

Tβ4 mRNA is expressed in developing mouth tooth germ, and it may play functional roles in the initiation, growth, and differentiation of tooth germ [12]. In addition, gene expression of DSPP, BSP, OCN, ON, and collagen type I related to mineralization is significantly decreased when Tβ4 is inhibited in the odontoblast-like cells MDPC-23 by Tβ4 siRNA [13]. Moreover, we recently reported that Tβ4-overexpressing transgenic mice promote abnormal hair growth and tooth development as observed by abnormally shaped white teeth and dull incisors [14]. Although Tβ4 peptide accelerates bone regeneration and osteogenesis of tooth extraction sockets [15], the underlying molecular mechanisms for controlling odontoblastic growth and differentiation by Tβ4 are still not fully understood in regenerative dentistry. The purpose of this study was to investigate the role of Tβ4 in odontoblastic differentiation of HDPCs and to identify the underlying signal transduction pathways involved.

## Materials and Methods

### Chemical and reagents

α-modified Eagle medium (MEM), fetal bovine serum (FBS), and other tissue culture reagents were purchased from Gibco BRL Co (Grand Island, NY). Tβ4 peptide purchased from Abcam (Cambridge, MA, USA). Lipofectamine 2000 was obtained from Invitrogen Life Technology (Grand Island, NY). The small interfering RNAs (siRNA) against ILK, antibodies to p-FAK, p-paxilin and ILK were purchased from Santa Cruz Biotechnology (Santa Cruz, CA). Antibodies against p-ERK, ERK, p-p38, p38, p-JNK, JNK, p-Smad1/5/8 and, p-Smad2/3 were purchased from Cell Signaling Technology (Beverly, MA). Antibodies for β-actin monoclonal antibodies and secondary antibodies and other chemicals were obtained from Sigma-Aldrich Chemical Co (St. Louis, MO).

### Cell culture

The immortalized HDPCs by transfection with the telomerase catalytic subunit of the human telomerase reverse transcriptase (hTERT) [16], were kindly provided by professor Takashi Takata (Hiroshima University, Japan). Cells were cultured in α-MEM supplemented with 10% FBS, 100 U/ml penicillin, and 100 µg/ml streptomycin in a humidified atmosphere of 5% CO_2_ at 37°C. For the induction of odontogenic differentiation, cells were cultured with osteogenic medium (OM; α-MEM supplemented with 10% FBS, 50 µg/mL ascorbic acid, 10 mM β-glycerophosphate and 100 nM dexamethasone) as described previously [17]–[19]. After cells reached 70% confluence, the experimental treatments were initiated. And then OM with Tβ4 siRNA or Tβ4 peptide was applied to cell culture for 7 or 14 days. The culture medium was replaced every 2 days during the incubation period. Our study was approved by the local ethics committee.

### Cell proliferation Assay

Cell proliferation was determined by viable cell counting. For cell number counting, the cells were cultured at 3 × 10^4^ cells per well in a 24-well culture plate. The number of viable cells after trypan blue exclusion was counted after 7 or 14 days of incubation at 37°C. Cell counts were performed in triplicate and repeated in five cultures (n = 5).

### Alkaline phosphatase Assay

HDPCs were plated in 6-well plates and incubated for 7 or 14 days in the same way as proliferation assay above. Treated cells were washed twice with ice-cold phosphate-buffered saline (PBS), then harvested in 1 ml 50 mM Tris–HCl (pH 7.6), sonicated twice on ice and then centrifuged at 4°C for 15 min at 1000×*g*. The supernatants were stored at −20°C until analysis for alkaline phosphatase activity was conducted, using *p*-nitrophenylphosphate as substrate. Absorbance was read at 405 nm using a microplate reader. Alkaline phosphatase activity was expressed as nM/well. The ALP assay was performed in triplicate and repeated in six cultures (n = 6).

### Alizarin Red S staining

After incubation in OM for 7 and 14 days, cell mineralization was determined using alizarin red S (ARS) staining. The cells were fixed in 70% ice-cold ethanol for 1 hour and rinsed with distilled water. Cells were then stained with 40 mM ARS (pH 4.2) for 10 minutes under conditions of gentle agitation. The pictures of ARS staining were photographed with a digital camera. Experiments were performed in triplicate wells and repeated at least three times.

### Tβ4 and ILK siRNA transfection

siRNA was used for transient gene knockdown studies. The HDPCs were transfected with double stranded Tβ4 or ILK siRNAs (30 nM) for 24 h using Lipofectamine 2000 (Gibco; Invitrogen Ltd, Paisley, UK) according to the manufacturer's instructions. Silencer Negative Control siRNA was used as a negative control and was introduced into the cells using the same protocol. After transfection, cells were cultured in six-well plates at 37°C until needed. The efficiency of gene knock down was evaluated by RT-PCR.

### RNA isolation and reverse transcriptase-polymerase chain reaction (RT-PCR)

The total RNA of cells was extracted using the Trizol reagent (Life Technologies, Gaithersburg, MD) according to the manufacturer's instruction. 1 µg of RNA isolated from each cultures was reverse transcribed using oligo (dT)^15^ primers (Roche Diagnostics, Mannheim, Germany) and AccuPower RT PreMix (Bioneer Corporation, Daejeon, South Korea). Thereafter, the RT-generated DNA (2–5 µl) was amplified. Primer sequences are detailed in Table 1. PCR products were subjected to electrophoresis on 1.5% agarose gels, stained with ethidium bromide. All assays were repeated 3 times to ensure reproducibility.

**Table 1:** Reverse transcriptase-polymerase chain reaction (RT-PCR) primers and conditions.

Genes	Primer Sequence (5′–3′)	Annealing emperature (°C)	Cycle umber	Product ize (bp)
Tβ4	F: 5′-CGCAGACCAGACTTCGCTCGTAC-3′	58	30	398
	R: 5′-TCCTTCCCTGCCAGCCAGATAGAT-3′			
ALP	F: 5′-ACGTGGCTAAGAATGTCATC-3′	55	30	475
	R: 5′-CTGGTAGGCGATGTCCTTA-3′			
OPN	F: 5′-CCAAGTAAGTCCAACGAAAG-3′	55	30	347
	R: 5′-GGTGATGTCCTCGTCTGTA-3′			
OCN	F: 5′-CATGAGAGCCCTCACA-3′	57	30	310
	R: 5′-AGAGCGACACCCTAGAC-3′			
DMP1	F: 5′-CAGGAGCACAGGAAAAGGAG-3′	56	36	213
	R: 5′-CTGGTGGTATCTTCCCCCAGGAG-3′			
DSPP	F: 5′-AGAAGGACCTGGCCAAAAAT-3′	60	35	280
	R: 5′-TCTCCTCGGCTACTGCTGTT-3′			
Runx2	F: 5′-AACCCACGAATGCACTATCCA-3′	62	30	76
	R: 5′-CGGACATACCGAGGGACCTG-3′			
Osterix	F: 5′-CTCTGCGGGACTCAACAACTCTG-3′	62	35	316
	R: 5′-GAGCCATAGGGGTGTGTCATGTC-3′			
BMP-2	F: 5′-CAATGGACGTGTCCCCGCGT-3′	65	30	365
	R: 5′-GCTGCCCTCTCCAACCGGTG-3′			
BMP-4	F: 5′-GCTCCGGCTGAGTATCTAGCTTGTC-3′	65	30	364
	R: 5′-AGCATGGCTCGCGCCTCCTAG-3′			
Integrin α1	F: 5′-TGCTGCTGGCTCCTCACTGTTGT-3′	65	35	703
	R: 5′-TAGTCTGGCGGCCACCTCTCTG-3′			
Integrin	F: 5′-TTTCCCTGCTCTCACCGGGC-3′	62	35	132
α2	R: 5′-ACCGGGGGACCGTAGTTGCG-3′			
Integrin	F: 5′-CCCATCCCTGATGCCCCCGT-3′	65	35	415
α3	R: 5′-TGCCCCCTCAGTAGTCGTCG-3′			
Integrin	F: 5′-GACGCCGCGCGGAAAAGATG-3′	65	35	159
β1	R: 5′-ACCACCCACAATTTGGCCCTGC-3′			
GAPDH	F: 5′-CGGAGTCAACGGATTTGGTCGTAT-3′	62	25	306
	R: 5′-AGCCTTCTCCATGGTGGTGAAGAC-3′			

### Western blotting

After treatment, cells (3 × 106 cells/in 60 mm dish) were collected and washed with phosphate-buffered saline (PBS). After centrifugation, cell lysis was carried out at 4°C by vigorous shaking for 15 min in RIPA buffer [150 mM NaCl, 1% NP-40, 0.5% sodium deoxycholate, 0.1% SDS, 50 mM Tris-HCl (pH 7.4), 50 mM glycerophosphate, 20 mM NaF, 20 mM EGTA, 1 mM DTT, 1 mM Na3VO4, and protease inhibitors]. After centrifugation at 14,800 g for 15 min, the supernatant was separated and stored at −70°C until use. The protein concentration was determined by using the BCA protein assay kit (Pierce, Rockford, IL, USA). After addition of sample loading buffer, protein samples were electrophoresed on a 12.5% SDS-polyacrylamide gel. Proteins were transferred to polyvinylidene difluoride membrane at 300 mA for 6 h. The blots were blocked for 1 h at room temperature in fresh blocking buffer (0.1% Tween 20 in Tris-buffered saline, pH 7.4, containing 5% non-fat dried milk). Dilutions (1∶1000) of primary antibodies were made in PBS with 3% non-fat dried milk. Following three washes with PBS-T (PBS and 0.1% Tween 20), the blots were incubated with horseradish peroxidase (HRP)-conjugated secondary antibodies in PBS with 3% non-fat dried milk for 1 h at room temperature. The blots were washed again three times in PBS-T buffer, and transferred proteins were incubated with ECL substrate solution (Amersham Pharmacia Biotech, Piscataway, NJ) for 1 min according to the manufacturer's instructions followed by visualization with X-ray film.

### Statistical analysis

Differences among groups were analyzed using one-way analysis of variance combined with the Bonferroni test. All values were expressed as means ± standard deviations and differences were considered significant at p<0.05.

## Results

### Time Course of Tβ4 mRNA and Protein Expression during Odontoblastic Differentiation of HDPCs

To investigate the expression of Tβ4 mRNA and protein during odontoblastic differentiation of HDPCs, cells were cultured in osteogenic medium (OM) for 14 days and the samples analyzed by conventional RT-PCR and Western blotting (Figure 1A). Expression of Tβ4 mRNA and Tβ4 protein was detected in unstimulated HDPCs and increased in a time-dependent manner following exposure to OM until 14 days after the initiation of treatment. The increase in Tβ4 protein expression in HDPCs correlated with a parallel increase in Tβ4 mRNA levels (Figure 1A).

**Figure 1:** Tβ4 mRNA and protein expression during odontoblastic differentiation of HDPCs. Cells were cultured in OM containing 10 mM β-glycerophosphate, 50 µg/ml ascorbic acid, and 100 nM dexamethasone for 0, 1, 3, 7 or 14 days. **(A)** Tβ4 mRNA expression was followed by RT-PCR relative to GAPDH expression (top) and by Western blotting relative to β-active expression (bottom). mRNA and protein expression of Tβ4 is upregulated during odontogenic differentiation in HDPCs. Effects of Tβ4 silencing on OM-induced growth and odontogenic differentiation of HDPCs **(B–F).** Cells were transiently transfected with Tβ4 siRNA (30 nM) for 24 h and then cultured in OM for 7 days. **(B)** Tβ4 knockdown by Tβ4 siRNA was detected by RT-PCR and Western blotting. **(C)** Cell proliferation was determined by viable cell counting (N = 5) for 7 days. Differentiation was assessed by **(D)** measuring ALP activity (N = 6), **(E)** RT-PCR, and **(F)** Alizarin Red staining for 7 days. Transfection with Tβ4 siRNA decreases OM-induced odontoblastic differentiation but not affected cell growth. ^*^ *P*<0.05 compared to the control; ^#^ *P*<0.05 compared with OM alone. Data are representative of three independent experiments.

### Effects of Tβ4 Silencing on OM-Induced Growth and Odontogenic Differentiation of HDPCs

HDPCs showed higher ALP activity, mRNA expression of the odontogenic differentiation genes, and mineralized nodule formation when cultured in OM compared with those in control medium, which results confirmed that HDPCs can differentiate into odontoblast-like cells (Fig. 1D–F). To examine the role of Tβ4 in OM-induced differentiation, Tβ4 expression in HDPCs was knocked down with a specific siRNA. As shown in Figure 1, Tβ4 siRNA successfully knocked down Tβ4 mRNA and protein expression in HPDCs (Figure 1B) and blocked OM-induced alkaline phosphatase (ALP) activity and mRNA expression of the odontogenic differentiation genes (ALP, OPN, OCN, DMP1, and DSPP), whereas transfection of cells with an equivalent amount of nonspecific siRNA had no effect (Figure 1B–E). In addition, Alizarin Red S (ARS) staining significantly decreased in Tβ4 siRNA-treated cells compared to that in untreated cells during differentiation (Figure 1F). In the presence of Tβ4 siRNA, cell proliferation was not affected compared to OM treatment (Figure 1C).

### Effects of Tβ4 Activation on Cell Growth and Odontogenic Differentiation of HDPCs

We next examined the effect of exogenous Tβ4 on growth and differentiation in HDPCs. In the presence of Tβ4 peptide, cell proliferation was not affected by OM treatment (Figure 2A). However, ALP activity, mRNA expression of differentiation markers such as ALP, OPN, OCN, DMP1, and DSPP, and mineralization nodule formation were markedly stimulated by Tβ4 peptide in dose- and time-dependent manners (Figure 2B–D).

**Figure 2:** Effects of Tβ4 activation on cell growth and odontogenic differentiation of HDPCs. Cells were treated with Tβ4 peptide in OM containing for 14 days. **(A)** Cell proliferation was determined by viable cell counting (N = 5). Differentiation was assessed by **(B)** measuring ALP activity (N = 6), **(C)** RT-PCR, and **(D)** Alizarin Red staining for 7 and 14 days. Tβ4 activation with a Tβ4 peptide promotes odontogenic differentiation, but not affects cell growth. ^*^ *P*<0.05 compared to the control; ^#^ *P*<0.05 compared with OM alone. Data are representative of three independent experiments.

### Effects of Tβ4 Activation on MAPK Pathways and Transcriptional Factors in HDPCs

To further explore the mechanistic basis underlying the differentiation potential of Tβ4-activated cells, we followed the expression and activation of the mitogen-activated protein kinase (MAPKs) p38, c-Jun N-terminal kinase (JNK), and extracellular signal-related kinase (ERK). OM treatment increased the phosphorylation, but not overall levels, of p38, JNK, and ERK (Figure 3A), and maximal expression of p38, JNK, and ERK was detected following incubation of HDPCs in OM for 120 min. Treatment with the Tβ4 peptide enhanced OM-induced phosphorylation of p38, JNK, and ERK, but had no effect on the overall protein levels.

**Figure 3:** Effects of Tβ4 activation on the expression of MAPK pathways and transcription factors in HDPCs. Cells were incubated without or with Tβ4 peptide (1 µg/ml) in OM. **(A)** Phosphorylation of p38, JNK, and ERK MAPK was determined by Western blot analysis for 180 min. **(B)** Expression of the transcription factors Runx2 and Osterix was examined by RT-PCR for 180 min. Tβ4 activation enhanced the phosphorylation of p38, JNK, and ERK, and expression of transcription factors such as Runx2 and osterix. Data are representative of three independent experiments.

We also examined whether Tβ4 peptide affected the expression of Runx2 and Osterix, transcription factors involved in osteoblast and odontoblast differentiation [20]. OM treatment significantly increased Runx2 and Osterix expression compared with the control (Figure 3B). Addition of Tβ4 peptide further upregulated Runx2 and Osterix mRNA expression in a time-dependent manner (Figure 3B).

### Effects of Tβ4 Activation on BMP pathway in HDPCs

To elucidate whether a BMP-dependent mechanism may be involved in Tβ4 activation of HDPCs, we examined BMP2 and BMP4 expression. mRNA expression of BMP2 and BMP4 was increased by Tβ4 peptide in time- and dose-dependent manner (Figure 4A). To determine whether Tβ4 activated signaling molecules downstream of BMP, Smad phosphorylation was examined. Tβ4 peptide significantly enhanced the phosphorylation of Smad1/5/8 and Smad2/3 in HDPCs compared with the OM treatment group (Figure 4B).

**Figure 4:** Effects of Tβ4 activation on BMP pathway in HDPCs. Cells were incubated **(A)** without or **(B)** with Tβ4 peptide in OM. **(A)** Expression of the BMP2 and BMP4 was examined by RT-PCR for 14 days. **(B)** Phosphorylation of Smad1/5/8 and Smad 2/3 was determined by Western blot analysis for 180 min. Tβ4 peptide increased expression of BMP2 and BMP4, phosphorylation of Smad1/5/8 and Smad2/3. Data are representative of three independent experiments.

Our preliminary and previous study [21] demonstrated that pretreated with a BMP-2 inhibitor noggin (1 µM) for 1 h blocked BMP pathway in HDPCs. Therefore, to exam whether Tβ4 peptide operated through a BMP-dependent pathway, cells were pretreated for 1 h with the BMP inhibitor noggin (1 µM) and then incubated with Tβ4 peptide (1 µg/ml) or BMP2 (100 ng/ml) for 14 days (Figure 5A–C) and 120 min (Figure 5D, E). The addition of noggin blocked BMP2- and Tβ4-induced ALP activity (Figure 5A) and mineralized nodule formation measured by ARS staining (Figure 5B). Pretreatment with noggin also abolished Tβ4 peptide-induced phosphorylation of Smad1/5/8 and Smad2/3 (Figure 5C), and phosphorylation of p38, JNK, and ERK (Figure 5D). Similarly, Tβ4-enhanced expression of Runx2 and Osterix mRNA was blocked by noggin (Figure 5E).

**Figure 5:** Effects of a BMP inhibitor on Tβ4 activation-induced odontogenic differentiation. **(A–C)** Cells were pretreated with noggin (1 µM) for 1 h, then incubated with Tβ4 (1 µg/ml) and BMP2 (100 ng/ml) for 14 days **(A–C)** or incubated for 180 min in OM **(D, E)**. Differentiation was assessed by **(A)** measuring ALP activity (N = 6) and **(B)** Alizarin Red staining for 14 days. Expression of **(C)** BMP2, BMP4, Smad, **(D)** MAPK, and **(E)** transcription factors were determined by RT-PCR and Western blot analysis for 180 min. Noggin blocked Tβ4 peptide-induced odontoblastic differentiation via Tβ4 peptide-induced phosphorylation of Smad1/5/8 and Smad2/3, and phosphorylation of MAPK and transcriptional factors. ^*^ *P*<0.05 compared to the control; ^#^ *P*<0.05 compared with OM alone. Data are representative of three independent experiments.

### Involvement of Integrin and Integrin-Mediated Signaling on Potentiating Effects of Tβ4 Activation in HDPCs

To examine the effects of Tβ4 activation on the expression of integrin signaling, we examined the expression of integrin subunits and downstream signaling molecules including phosphorylated focal adhesion kinase (p-FAK), p-paxillin, and integrin-linked kinase (ILK), which have been previously shown to be stimulated by Tβ4 in cardiomyocytes [22]. Analysis by RT-PCR revealed that Tβ4 upregulated integrin α1, α2, α3, and β1 mRNA in a dose- and time- dependent manner (Figure 6A). Phosphorylation of paxillin and FAK increased with time 0–180 min in cells treated with OM, but the effect was markedly greater at 90–180 min in cells exposed to Tβ4 (Figure 6B). In addition, ILK levels in Tβ4 treated cells were higher than in comparable cells grown in OM.

**Figure 6:** Involvement of integrin and integrin-mediated signaling on effects of Tβ4 activation in HDPCs. Cells were incubated **(A)** without or **(B)** with Tβ4 peptide in OM. Expression of integrin (A) and its downstream signaling molecules (B) were determined by RT-PCR and Western blot analysis for 180 min and 14 days, respectively. The expression of integrin and its downstream signaling molecules including p-FAK, p-paxillin, and ILK were increased by Tβ4 peptide. Data are representative of three independent experiments.

To further elucidate whether the activation of ILK was necessary for the odontoblastic differentiation inducing effects of Tβ4, ILK-specific siRNAs were used to knock down ILK. ILK silencing inhibited Tβ4-induced ALP activity (Figure 7A) and mineralized nodule formation (Figure 7B). Furthermore, transfection of HDPCs with ILK siRNA abolished Tβ4 peptide-mediated activation of BMP signaling, including phosphorylation of Smad1/5/8, Smad2/3 (Figure 7C), and MAPK signaling, including phosphorylation of p38, JNK, and ERK (Figure 7D). Similarly, Tβ4-enhanced expression of Runx2 and Osterix mRNA was blocked by ILK siRNA (Figure 7E).

**Figure 7:** Effects of ILK silencing on Tβ4 activation-induced odontogenic differentiation of HDPCs. Cells were transiently transfected with ILK siRNA (30 nM) for 24 h and then cultured in OM for 7 days **(A–C)** or incubated for 180 min in OM **(D, E)**. Differentiation was assessed by **(A)** measuring ALP activity (N = 6) and **(B)** Alizarin Red staining for 7 days. Expression of **(C)** BMP2, BMP4, Smad, **(D)** MAPK, and **(E)** transcription factors were determined by RT-PCR and Western blot analysis for 180 min. ILK siRNA blocked Tβ4-induced odontoblastic differentiation, and activation of the BMP, MAPK, and transcription factor pathways. ^*^ *P*<0.05 compared to the control; ^#^ *P*<0.05 compared with OM alone. Data are representative of three independent experiments.

## Discussion

Operative dentistry has attempted to use some regenerative approaches [e.g., the use of mineral trioxide aggregate (MTA) and Ca(OH)_2_ for vital pulp therapy] to stimulate reparative or reactionary dentine, but the outcome has not always been predictable. Current evidence suggests that the implantation of external signaling molecules in the exposed pulp can induce the formation of a reparative dentinal bridge in the coronal pulp, where cells implicated in the reparative process are recruited, proliferate, and differentiate into osteoblast-like and odontoblast-like cells [23]. Multiple signaling molecules, such as BMPs, fibroblast growth factors (FGFs), Sonic hedgehog, and Wnt proteins, have been implicated as mediators of these tissue interactions [22]. In addition, the transforming growth factor (TGF)-β family and BMPs are important in cellular signaling pathways mediating odontoblast differentiation and stimulation of dentine matrix secretion and are hence essential for pulp regeneration [24], [25]. Previously, we reported that recombinant human FGF-2 (rh-FGF-2), rh-dentin sialoprotein, mineral trioxide aggregate (MTA), MTA plus enamel matrix derivative, simvastatin, Portland cement (PC), bismuth-oxide containing PC, calcium phosphate cement, and mechanical stress promoted growth and odontoblastic differentiation in HDPCs [21], [26]–[31]. Moreover, we demonstrated that heme oxygenase-1, lysyl oxidase, and SIRT1 are novel molecular targets of HDPC differentiation and may have clinical implications for regenerative endodontics [32]–[34]. Although Tβ4 is expressed in developing mouth tooth germ [12], its role is not well defined in pulpal regeneration. In this study, we investigated whether Tβ4 plays a role in odontoblastic differentiation. To our knowledge, this is the first reported study examining the expression of Tβ4 during odontoblastic differentiation, the effects of activating Tβ4 with peptide, and inhibiting it using Tβ4 siRNA, on the growth and differentiation of HDPCs.

In the present study, Tβ4 mRNA and protein were time-dependently increased throughout the entire HDPC differentiation process. This result differs from that in a study on MDPC-23 cells [13], which showed that Tβ4 mRNA and protein was strongly increased after 4 days and decreased from 14 to 28 days during differentiation of MDPC-23 cells, which might be related to differences in cell types or species and culture conditions.

ALP is expressed at the early stages of both osteoblast and odontoblast differentiation, providing an inorganic phosphate for hydroxyapatite formation [35]. ON, OPN, OCN, and DMP1 function as modulators of the formation and growth of hydroxyapatite during mineralization [36]. DSPP is considered a terminal phenotypic marker of mature odontoblasts [37]. To assess the role of Tβ4 in HDPC odontoblastic differentiation, we evaluated the effects of Tβ4 inhibition and activation on the expression of key differentiation markers. Our results indicate that inhibition of Tβ4 by siRNA in HDPCs decreased ALP activity, mineralized nodule formation, and upregulated the expression of mRNAs encoding odontoblastic markers, including ON, OPN, OCN, DSPP, and DMP1. These results are consistent with previous data obtained using the odontoblast-like cells MDPC-23 [13]. Furthermore, activation of Tβ4 by exogenously added Tβ4 peptide in HDPCs increased OM-induced odontoblastic differentiation in a dose-dependent manner. Our results suggest that odontoblastic differentiation is promoted by Tβ4 activation and suppressed by Tβ4 inhibition. Thus, the differentiation of HDPCs into odontoblasts appears to be controlled, at least in part, by a Tβ4-dependent mechanism.

We next investigated whether Tβ4 influenced the phosphorylation of kinases because activation of MAPKs, including p38, JNK, and ERK, has been reported to contribute to odontoblastic differentiation in HDPCs [27], [29]. In this study, OM-induced phosphorylation of p38, JNK, and ERK was significantly enhanced by Tβ4 peptide (Fig. 3A). In oligodendrocyte differentiation, Tβ4 peptide treatment upregulates p38 MAPK [38], and the activation of ERK by Tβ4 in endothelial progenitor cells has been reported [39]. These conflicting observations may result from differences in experimental procedure, cell type, or stimuli.

Odontoblast differentiation is tightly coordinated by the activities of transcriptional regulators. These include the master transcription factors Runx2 and Osterix, which govern the expression of genes involved in the developmental process [20]. In the present study, we investigated the expression of Runx2 and Osterix and demonstrated that Runx2 and Osterix increased with Tβ4 induction time. Consistent with the results examining ALP activity and mineralization, the expression of Runx2 and Osterix was much higher with Tβ4 treatment than in OM.

BMP signaling is initiated by receptor binding, propagated by the phosphorylation of the Smad1/5/8 complex, and finally translocated into the nucleus, resulting in the regulation of target gene transcription [40], [41]. Noggin is one of the osteoblast-secreted proteins that can limit BMP signaling by interacting with BMP, thereby preventing receptor binding [42]. Previous studies reported that Smad1/5 is involved in BMP-2-induced odontoblastic differentiation in DPCs [43]. In this study, we found that Tβ4 peptide enhanced the expression of BMP2 and BMP4 mRNA, and its downstream molecule Smad1/5/8 and Smad2/3 protein, suggesting that Tβ4 influences HDPC functions through the BMP pathway. This finding was further supported by the fact that noggin blocked Tβ4-induced ALP activity, mineralized nodule formation, and activation of Smad1/5/8, Smad2/3, p-38, JNK, ERK, Runx2, and Osterix. Thus, the BMP pathway is critical for Tβ4-mediated odontoblastic differentiation of HDPCs.

Matrix responsiveness during osteogenesis is caused by the aggregation of the α2β1 and αvβ3 integrins that subsequently activate intracellular signaling cascades including paxillin, FAK, and ERK/MAPK pathways, resulting in the phosphorylation of the osteoblast-specific transcription factor Osterix/Runx2 [44], [45]. In the present study, the integrins α1, α2, α3, and β1 were highly expressed in HDPCs exposed to Tβ4. Phosphorylated paxillin, phosphorylated FAK, and ILK were also found at elevated levels in Tβ4 treated HDPCs. Cell–extracellular matrix interactions can activate ILK, which interacts with the cytoplasmic domain of both β1 and β3 integrins [46]. The current study showed that ILK silencing inhibited subsequent Tβ4-induced odontoblastic differentiation. Furthermore, ILK siRNA antagonized Tβ4-induced Smad1/5/8, Smad2/3, p-38, JNK, ERK, Runx2, and Osterix expression. Thus, these results suggest that Tβ4 promotes odontoblastic differentiation in cultured HDPCs via the integrin/ILK/BMP signaling pathway.

In conclusion, our present study is the first to demonstrate that HDPC odontoblastic differentiation is activated by Tβ4 induction and attenuated by Tβ4 inhibition via p38, JNK, ERK, BMP, and integrin pathways. Thus, Tβ4 may be a new therapeutic target for regenerative endodontics. Further elucidation of the role of Tβ4 as bioactive agents for pulp repair or tissue engineering is necessary.
